# Classification of COVID-19 and Pneumonia Using Deep Transfer Learning

**DOI:** 10.1155/2021/3514821

**Published:** 2021-12-16

**Authors:** Mainuzzaman Mahin, Sajid Tonmoy, Rufaed Islam, Tahia Tazin, Mohammad Monirujjaman Khan, Sami Bourouis

**Affiliations:** ^1^Department of Electrical and Computer Engineering, North South University, Bashundhara, Dhaka 1229, Bangladesh; ^2^Department of Information Technology, College of Computers and Information Technology, Taif University, P.O. Box 11099, Taif 21944, Saudi Arabia

## Abstract

The World Health Organization (WHO) recognized COVID-19 as the cause of a global pandemic in 2019. COVID-19 is caused by SARS-CoV-2, which was identified in China in late December 2019 and is indeed referred to as the severe acute respiratory syndrome coronavirus-2. The whole globe was hit within several months. As millions of individuals around the world are infected with COVID-19, it has become a global health concern. The disease is usually contagious, and those who are infected can quickly pass it on to others with whom they come into contact. As a result, monitoring is an effective way to stop the virus from spreading further. Another disease caused by a virus similar to COVID-19 is pneumonia. The severity of pneumonia can range from minor to life-threatening. This is particularly hazardous for children, people over 65 years of age, and those with health problems or immune systems that are affected. In this paper, we have classified COVID-19 and pneumonia using deep transfer learning. Because there has been extensive research on this subject, the developed method concentrates on boosting precision and employs a transfer learning technique as well as a model that is custom-made. Different pretrained deep convolutional neural network (CNN) models were used to extract deep features. The classification accuracy was used to measure performance to a great extent. According to the findings of this study, deep transfer learning can detect COVID-19 and pneumonia from CXR images. Pretrained customized models such as MobileNetV2 had a 98% accuracy, InceptionV3 had a 96.92% accuracy, EffNet threshold had a 94.95% accuracy, and VGG19 had a 92.82% accuracy. MobileNetV2 has the best accuracy of all of these models.

## 1. Introduction

Pneumonia (lung infection) is an acute pulmonary disease. It is an inflammatory condition typically induced by pathogens, physicochemical causes, immunological injuries, and other pharmacological agents. There are many prominent approaches to classifying pneumonia. Contagious as well as noninfectious pneumonia is categorized as infectious based on different pathogens, in which case pneumonia is then categorized as being caused by bacteria, viruses, mycoplasmas, chlamydial pneumonia, and so forth. Noninfectious pneumonia and aspiration pneumonia caused by physical, chemical, and radiation pneumonia are categorized as innate immunity pneumonia. Pneumonia is categorized as CAPs based on several diseases, of which CAP is a greater proportion (community-acquired pneumonia), HAP (hospital-acquired pneumonia), and VAPs (ventilator-associated pneumonia). The diverse range of infections makes HAP more resistant to various antibiotics and easier to grow, which makes therapy harder [1]. On the other hand, on December 31, 2019, the World Health Organization received a report of a group of unidentified pneumonia cases in Wuhan, Hubei Province, China. An unknown new virus has been detected in January 2020 [2, 3]. A very regrettable coronavirus pandemic (COVID-19) appears to be the second wave that is more hazardous than the first wave. In terms of the second wave of COVID-19, India is among the most affected regions in the world. The United States and Brazil are two nations also susceptible since they did not recover from the very first wave. The number of affected individuals was 360,960 in India on April 26, 2021, and is quickly growing [4]. For Bangladesh, this is concerning because of its near geographic position, and the Indian variant is more hazardous than other variations around the world. The virus is increasingly growing and therefore can be caught at any age, leading to severe diseases.

Both pneumonia and COVID-19 are deadly to human beings. Over 800,000 children under five per year are killed by pneumonia, and around 2,200 die every day. Over 1,400 children per 100,000 children are afflicted with pneumonia [5]. The latest study found that the foremost cause of mortality was lower respiratory tract illness, particularly pneumonia, in 2013. In Indian countries, the most pneumonia fatalities in India were reported in the current John Hopkins Bloomberg School of Public Health, and in 2015, there were something like 0.297 million pneumonia deaths and deaths from dysentery in children under the age of 5. In 2015, pneumonia was also the world's number one killer of children under age 5 [6]. Besides pneumonia, the infection rate of COVID-19 is pretty high. COVID-19 is a very infectious viral illness caused by SARS-CoV-2 and is the largest pandemic throughout the globe since the 1918 influenza outbreak that killed more than 2.9 million people worldwide. The risk of SARS-CoV-2 infection should be increased for those over 60, including those with health issues. One problem that has been determined is that both pneumonia and coronavirus have adverse impacts on the health of the lungs. Hence, doctors encourage patients to use an oxygen analyzer to keep track of their oxygen consumption in order to discover and correct any irregularities as soon as feasible. CNNs are suitable to address this sort of problem [7].

In the human body, these viruses target the palm and, in extreme situations, lead to pneumonia. It reduces the amount of oxygen instantly thereafter. In the case of COVID-19, it is different. Since coronavirus does not have treatment up to now, preventing transmission of the virus is the sole approach before any vaccination. The first and only options to date are tests and traces. With technology development, more and more metrics in which radiology-based techniques are most preferred, and most beneficial are being created. The diagnostic radiology methods for lung illness include thoracic X-ray imaging, CT, and MRI, which are thoroughly effective and cost-effective chest X-ray imaging methods, as well as accessible in hospitals, and have reduced dosage exposures to individuals.

But the identification of pneumonia and COVID-19 with X-ray images is still an enormous job, even for skilled and experienced clinicians, as X-ray photos provide comparable location features for other illnesses, including lung disease. Another test is PCR, also known as a polymerase chain reaction, which is impossible due to the rapid increase in the number of instances. Alternate diagnostics are thus necessary to swiftly identify, quarantine, or separate sick people. By far, deep transfer learning techniques for the identification of viruses have indeed been employed. The outcomes of such deep learning approaches, though, will not be enough to address the medical diagnostic procedure.

This study offers a profound learning method for the identification of patients with SARS-CoV-2. Feature extraction with excellent performance may be accomplished in the classification in the CNN model. The CNN model uses filter-based extraction features, which may be effectively classified. CNNs can categorize complicated identity pictures. Deep transfer learning will be used to decrease a large number of weight factors. This article claims that COVID-19 and pneumonia will be classified in depth. CT scan images, specifically CXR images, were chosen as a test data set in this study because X-ray equipment is low-cost, time-effective, and compact in almost all clinics. This study can thus assist fewer underdeveloped nations. In the quickest possible time, this approach will assist in discovering the coronavirus and pneumonia from CXR pictures. Chest x-rays are among the most popular radiology exams. CXR evaluation includes thoracic disease identification and location. A variety of papers related to the algorithm, COVID-19, and pneumonia were read. Artificial intelligence (AI) has been used in a variety of fields (e.g., illness diagnosis in healthcare) [8–10]. Perhaps one of AI's key benefits is that it may be used for the classification of unobserved pictures in a training set. In this work, AI was applied to determine if a patient's chest X-ray picture is COVID-19 affirmative. Two key themes [11] were highlighted by Wynants et al. The initial idea included research on COVID-19 detection as well as research on the prediction of the number of individuals affected in the next couple of days. The investigation showed that almost all of the models currently available are inadequate and partial. In order to stimulate more specific detection and modelling techniques, analysis data on COVID-19 should be made available to the public.

Redmon et al. [12] presented YOLO in 2016, which eliminates the need for a separate area proposal network and allows for detection speeds of up to 45 frames per second. The SSD algorithm was introduced by Liu et al. [13] in the same year. In terms of detecting speed, all SSD and YOLO win, but SSD employs a multiscale feature map to recognize separate. The spatial resolution of deep networks' images has been substantially reduced, making it harder to locate small targets that are hard to detect at low resolution, lowering detection accuracy. For standalone diagnosis, YOLO does not use multiscale feature maps. It helps smooth the extracted features and clip them with a lower-resolution feature map, but it only treats diagnosis as a regression problem, which results in low detection accuracy. Girshick et al. introduced R-CNN in 2014, which increased training speed considerably. In the PASCAL VOC 2010 sample, the mAP increased from 35.1% to 53.7%. Ren and colleagues introduced the Faster R-CNN method in 2015, which uses RPN to generate feature map recommendations (region proposal network). DetNet was introduced by Lee et al. [14] in 2018, and it was developed specifically for target detection, producing better detection results with fewer layers. The network uses a low-complexity expanded bottleneck structure to overcome the high computational complexity and memory usage induced by the high-resolution feature map; a higher feature map resolution is secured, while a higher subtractive field is achieved. To investigate pneumonia prediction, this study uses the DetNet concept and the Faster R-CNN framework.

In numerous areas, such as malware detection [15–18], mobile malware diagnosis [19–22], healthcare [23–25], and data recovery [26–30], people regularly use machine learning. It keeps increasing. An advanced ML structure called deep learning focused on a convolutional neural network (CNN) was created in 2012. It managed to win the world's most renowned computer-vision contest for the classification of ImageNet [31]. Deep learning algorithms allow data recognition at many levels of abstraction in computer models made up of a number of processing layers upon layers. Those who explicitly train a computer model to perform classification tasks based on images, writings, or sounds. Deep learning models, according to LeCun et al. [32], offer high precision and, in some cases, can promote better output. A ResNet50-based CNN with transfer learning utilizing ImageNet parameters was able to detect COVID-19 with 94% accuracy [33] against a respectable degree of CT slice using an unspecified lot of international data sets as a corpus. Many experts have been studying methods to detect pneumonia in recent times. To detect chest X-ray irregularities, Abiyev and Ma'aitah [34] use a convolutional neural network (CNN). CNN is more reliable than back-propagation neural networks (BPNN) and recurrent neural networks (RNN) while taking longer to train. To diagnose pneumonia in chest X-ray pictures, Vijendran and Dubey [35] utilize a combination of multilayer extreme learning machines (MLELM) and online sequential extreme learning machines (OSELM). On a data set of approximately 600 radiographs, Abiyev and Ma'aitahan examine the attributes retrieved from CNN layers as well as a set of conventional characteristics such as GIST and bag of words.

Although prior algorithms were executed fine in the diagnosis of pneumonia, the quantity and size of the data engaged were not enormous, and other academics conducted research on the deep network utilizing a substantial amount of data. On the RSNA (Radiological Society of North America) data set, Jaiswal et al. [36] used Mask R-CNN to predict probable pneumonia, and the intersection over union-based mAP was 21.8%. To overcome the chest X-ray data set's difficulty, Guendel et al. [37] suggested using DenseNet. Chakraborty et al. [38] designed a 17-layer convolutional neural network architecture with a large number of dense layers. On a data set of chest X-rays, it has an AP of 95.62%. Wang et al. [39] employed a deep convolutional neural network to incorporate a unified weakly supervised multilabel picture categorization and illness localization framework to overcome the limitations of ChestX-ray8. These tactics have been changed to meet the topology of the network, but not for backbone upgrades. It is essential to have a backbone built specifically for detection. In recent years, several approaches, including some deep learning algorithms, have been proposed to explain a quick procedure in pneumonia identification utilizing chest X-ray pictures. Deep learning has been used to improve the performance of computer-assisted diagnosis (CAD), particularly in the fields of medical imaging [40], picture segmentation [41, 42], and image reconstruction [43, 44]. Rajpurkar et al. [45] introduced DenseNet-121 [46], a 121-layer CNN model, in 2017 to speed up pneumonia diagnosis. The framework received a better F1 score than experienced doctors. Furthermore, in order to mitigate the effect of unbalanced classes, the researchers developed weighted binary cross-entropy loss, which differed from binary cross-entropy loss in that it assigned various weights to imbalanced classes based on their number.

The suggested loss, on the other hand, took into consideration the various training difficulty levels of the classes. Liang and Zheng [47] utilized residual connection networks [48] and dilated convolution [49] in the backbone network model to overcome the problems of poor generalization ability caused by overfitting and the problem of spatial sparseness produced by conventional convolution operations. Their model's overall recall rate and F1 score were 96.7% and 92.7%, respectively. The CNN approach developed by Jain et al. [50] coupled with transfer learning successfully utilized image characteristics learnt in a large data set, sped up the model's training process, and made it more difficult for the network to fall into local minimum points. In addition, two training models were proposed. Furthermore, the data set utilized by Jain et al. came from Kaggle, a well-known organization and competition site that hosts a variety of events and draws dedicated competitors looking to improve their ranking. The data set is separated into three subsets: training, validation, and testing. The validation subset is utilized to change the model's parameters, whereas the training subset is utilized to train the model. The testing subset is used to verify the model's generalization ability. In [51], to predict Alzheimer's disease, different ML algorithms have been used. Authors in [52] used CNN to detect COVID-19 from a chest X-ray. Different techniques have been used for COVID-19 detection in [53, 54].

The majority of studies, including chest X-ray imaging, have demonstrated an accuracy of 90–94%. Using X-ray images of the chest, the main objective of this research is to train pretrained models for transfer learning. A novel aspect of our study is the fact that we changed the parameters of MobileNetV2 and attained the greatest accuracy (98%), VGG19 (92.82%), Inceptionv3 (96.92%), and EffNet Threshold (94.95%). Deep learning may be used to identify COVID-19 and pneumonia, according to new research. To solve this sort of problem, convolutional neural networking, or CNN, is an excellent choice.

As previously stated, the major contribution of this study is the implementation of four distinct transfer learning algorithms on a freely accessible data set. Everything that came out of the implementation process was covered in the section devoted to findings and analysis.

The remainder of the manuscript is organized in the following manner.  Section 2 is devoted to discussing the materials and methodology. Obtained results are presented in Section 3. The conclusion part is finally delivered in Section 4.

## 2. Materials and Methodology

The data was gathered from open-source websites such as Kaggle. The data sets contain chest X-ray images from patients with pneumonia and COVID-19. A CNN is used to extract features. Four conv2D layers, three Maxpooling2D layers, one flatten layer, two dense layers, and a ReLU activation function are all included in the model. Softmax, the final thick layer, serves as an activation function.

The accuracy of the produced model is compared to the accuracy of the pretrained model in this research using transfer learning. MobileNetV2 was used for pretrained models, with slight changes in the last layers, and was prepared ahead of the basic model. Average pooling, Flatten, Dense, and Dropout are the customizable final layers. When it comes to extracting visual information, the CNN model excels. The algorithm extracts the attributes of the provided photographs and learns and distinguishes them using these qualities.

### 2.1. Software Tools and Materials

For data analysis, Python is the preferred programming language. Deep-learning-based problems could be solved using Python programming. A personal GPU is required to cope with data set preparation. Anaconda Navigator and Jupyter Notebook and other tools were used to implement and evaluate the proposed method. Any GPU's data, code, and work can be recovered via Git.

### 2.2. Description of the Data Set

Scans of chest X-ray images from two classes are included in the collection. COVID-19 patients' chest X-ray images are kept in one class, whereas pneumonia patients' images are kept in another. These categories are further broken into two categories. The first is a training set, while the second is a validation set. The COVID-19 patient's chest X-ray has 1,142 images, while the pneumonia patient's chest X-ray has 4,237 images [55]. For this investigation, the data set is divided into training (70%), testing (20%), and validation sets (10%). Data augmentation has been used to increase data diversity without having to collect new data. Figures 1 and 2 show the COVID-19 and the pneumonia patient's chest X-rays, respectively.

Figures 1 and 2 show a COVID-19 affected chest X-ray picture and a pneumonia chest X-ray image, respectively. The pictures in the collection have varying heights and widths when they are first created. In the model, the form of the provided pictures has been fixed.

### 2.3. Block Diagram

The chest X-ray image of a data set containing two subsections: COVID-19 patients and pneumonia patients are provided as input in Figure 3. This system starts with some preprocessing steps before performing the fitting task. These preprocessing steps are mainly importing photos, splitting data sets, and applying the data augmentation process. Fitting and fine-tuning the model resulted in increased precision. The confusion matrix, model loss, and model accuracy have been used to display the path that leads to how loss and accuracy fluctuate with epoch. Finally, if a user submits an image as an input model, the output section may detect whether the image is a COVID-19 patient image or a pneumonia image. The whole system is depicted most simply in the block diagram. This system's decision-making component is important, and it plays an important role in this research. The model, which was trained with a vast quantity of data taken from chest X-ray scans, is primarily responsible for the choice.

The complete system is presented in the simplest possible way in the block diagram. This system's decision-making component is critical. The decision is made mostly by the proposed model.

### 2.4. System Architecture

A CXR representation is placed into the system with this design, and the result is an illustrated forecast. It will determine if the picture is COVID-19 and pneumonia impacted in this situation. There are three streams, and the input shape is 224 × 224. Our design involves a filter size of 32 for padding, a kernel size of 3, and an activation function based on ReLU for the two first layers. The first max-pooling layer has a pool size of 2 and strides of 2. The further plain layer combines all of the pooled characteristics into a separate cell. In the end, two thick layers were produced. The activation function for the first layer is ReLU, while the activation function for the least thick layer is softmax. The features are added to the network once they have been preprocessed. A bird's-eye perspective of the structure is shown in Figure 4.

#### 2.4.1. Convolutional Layer

Deep transfer learning's basis is the convolutional layer. This group is in charge of deciding on design elements. A filter is applied to the source picture in this layer. Convoluting the results of the same filters yields the function map. The input is multiplied using a convolution process, which conducts the multiplication of weight ranges. A filter is created by multiplying an array of input data with a two-dimensional set of weights. When applied to a filter-sized patch of the source and the filter, a dot product gives a single value. Between the input's filter-sized patchwork and the filter, this product is utilized. The filter has a narrower range than the input and is utilized to multiplex data from numerous sources with the same filter. The filter is designed as a unique way of recognizing particular kinds of features since it carefully encompasses the whole frame.

Suppose the XX input is VRJK, with *J* indicating the features of the input frequency band and *K* denoting the cumulative set of input bandwidths. In the particular instance of filter bank attributes, *K* refers to the size of the filter bank function vector. Assume that *v*=[*v*_1_, *v*_2_,…*v*_*K*_], where *v*_*K*_ is the band *b* function vector. The following formula can be used to calculate the activations of the convolution layer:

(1) $$\begin{array}{c} g_{d,e}=\;\theta \left(\sum_{b=1}^{s}w_{b,d}^{T}v_{b+e-1}+a_{d}\right), \end{array}$$

where *g*_*d*,*e*_ is the *d*^th^ feature map's bias, which is the output of convolution layer of *e*^th^; *s* specifies the filter scale; *w*_*b*,*c*_ is the weight of the *d*^th^ filter; *a*_*d*_ is the *c*^th^ feature map's bias; and (*x*) stands for the activation function [57].

By allowing feature downsampling, the pooling layer highlights the availability of features. This has some spatiotemporal invariance and is mainly attributed to a convolution layer. The average presence and the maximum active occurrence of a function are represented by both average pooling and max pooling, respectively [58].

The pooling layer, in effect, removes superfluous characteristics from the pictures and renders them readable. Each time the layer averages the significance of its current stance, this is known as “average pooling.” When max pooling is used, the layer chooses the largest value from the current view of the filter each time. The max-pooling approach chooses just the highest value using the matrix size provided for each feature map, leading to fewer output units. As a result, the image shrinks dramatically, but the context stays the same. To avoid overfitting, a dropout layer is employed, and a pooling layer is employed to limit the number of feature mappings and system parameters. The following formula can be used to compute the activation of max pooling:

(2) $$\begin{array}{c} a_{b,c}=\;\max_{d=1}^{r}\left(h_{b,\left(c-1\right)\left(n+d\right)}\right), \end{array}$$

where *a*_*b*,*c*_ is the performance of the pooling layer, *n* denotes the subsampling factor, *r* denotes the pooling scale, and *n* denotes the subsampling factor.

#### 2.4.2. Flatten Layer

In this context, we investigate the flattened layer to transform data as a 1D array to generate a single long and narrow 1D feature vector. Vectors can be flattened if desired. Furthermore, it links the single vector to the final classification model, creating a completely linked layer [59]. All pixel data is included in a single layer that is fully linked. The last phases of deep transfer learning are flattened and completely linked layers. It is converted into a one-dimensional array in preparation for the next completely connected layer of photo classification.

#### 2.4.3. Fully Connected Layer

Fully connected layers are used a lot in deep transfer learning, and they have been shown to be quite effective in computer vision for picture identification and detection. The deep transfer learning method begins with convolution and pooling, which divides the picture into characteristics and analyses each one independently [60].

Every input is linked to all the neurons in a fully connected layer, and the inputs are flattened. As a completely linked layer, the ReLU activation function is frequently employed. In the final layer of the completely linked layer, the softmax activation function was used to estimate the output visuals. A fully connected layer is used in the convolutional neural network architecture. These are the final and most important layers of a convolutional neural network. This architecture makes use of a fully connected one.

#### 2.4.4. Pretrained Models

One of the most critical challenges for academics in healthcare research is a lack of medical records or data sets. Both time and money are spent on data processing and labelling. The benefit of transfer learning is that it eliminates the requirement for big data sets. Simulations are becoming more straightforward. Transfer learning is a method of transferring a formerly trained model from a big data set to a new model that must be trained with less data. This method began by training deep learning techniques using a small data set for a specific task, then adding a big-scale data set that had previously been trained in the training data set models [61].

In this research, three deep transfer learning-based pretrained models were utilized to categorize CXR images. The models utilized were MobileNetV2, VGG-16, and InceptionV3. CXR images were divided into two categories. One is in good health, whereas the other has SARS-CoV-2 and pneumonia. In addition, this research utilized a transfer learning method that employs ImageNet data to perform well with minimal data and is easy to train.  Figure 5 depicts the transfer-learning approach's symmetric system architecture.

The architecture of the system is divided into four components, as stated in Figure 5. The two first steps are selecting and inputting images and applying the pretrained model, respectively. Three pretrained models are loaded in the second stage. In the third segment, the layers shown in Figure 5 were used to change the loaded pretrained models. Finally, in the output portion, the findings will be given as COVID-19 and pneumonia infected and uninfected patients.

Over a range of model sizes, MobileNetV2 increases the cutting-edge efficiency of flexible models on a range of assignments and seat stamps. In each line, MobileNetV2 works as a chain of *n* repeating layers [62]. To factorize the regular state into depth-wise convolution, MobileNet employs depth-wise separable. Referring to [63], an 11-depth convolution, also called a point-wise convolution, is also employed. Another pretrained algorithm that was employed was InceptionV3. It has a maximum number of pooling layers in most scenarios. VGG16 is very useful because of its ability to extract features using a tiny kernel at low concentrations. The attributes of CXR images can be effectively obtained by a compact kernel [64].

## 3. Result and Analysis

Several network designs were tested throughout the selection process, including VGG-19, InceptionV3, EfficientNet, and MobileNetV2. A bespoke 19-layer ConvNet is also tried, but the network does not function well. TheMobileNetV2 has outperformed all other networks, and the findings based on that design are included.  Table 1 shows the accuracy and loss of four explored models over time. VGG-19 had the lowest accuracy of all the models (92.82%), whereas MobileNetV2 had the best accuracy (98%).

### 3.1. Model Accuracy

With the history of accuracy, everyone can see that the accuracy of the train is quickly increasing after every epoch. The accuracy in the first epoch was 89.5%, and then it increased in every epoch. In contrast, the model's validation accuracy was 89%, and it improved till the last epoch. During this period, it could be seen from the plot of model accuracy that a growing line was drafted for the accuracy of the train and for the test accuracy of about 91–96%. Figures 6–8 show the model accuracy, model loss, and model AUC, respectively.

Figure 7 shows that the validation loss is greater than the training loss. It also proves that our model is not overfitted. In the beginning, the validation and training loss was close to 0.3%, but at the end, the loss decreased for each of the epochs.

The system's confusion matrix is shown, with real values in columns and expected values in rows. The confusion matrix is a summary of the prediction results in a classification model. The correct and incorrect predictions from the confusion matrix are summarized and categorized.  Figure 9 illustrates the confusion matrix.

Figure 9 shows that this model can predict 527 images correctly and 13 images incorrectly. Predictions, data, and features are all crucial in error analysis. In a prediction-based error analysis, a confusion matrix can be utilized to represent the percentages of true positives, true negatives, false positives, and false negatives. The error analysis is also influenced by the size and nature of the data. Because the training and test sets can have a large impact on the outcome, properly separating the data for training and testing is equally critical for error analysis. In error analysis, features are extremely important. To eliminate errors, feature engineering and regularization were also used.

### 3.2. Model Test

The model was also subjected to real-world testing by using chest X-ray pictures as input. For this research, four output hdf5 files were generated. For the test, a new notebook file with the ipynb extension is created. Individual chest X-ray photographs were provided as input to the test file, which incorporated four models. The results of the test are presented in Figure 10, along with a prognosis of whether it is COVID-19 or pneumonia.

The model was fed a SARS-CoV-2-affected CXR image in Figure 10. The model then gave its output, which was a COVID-19 patient CXR image. Following this test, the model was fed another CXR image, which was pneumonia. The results of the standard CXR image are shown in Figure 11.

Figure 11 depicts a pneumonia output, and this image depicts a pneumonia-affected person, indicating that the model correctly anticipated the patient's condition. This examination included not only these two experiments but also all possible models.

### 3.3. Model Comparison

The VGG19, InceptionV3, and MobileNetv2 pretrained models in this study were compared to various previous models. In this investigation, InceptionV3, MobileNetV2, and VGG19 produced higher outcomes, accuracy, and efficiency than the models in the relevant studies. The accuracy of the pretrained models grew significantly. The comparison of different models and data sets is shown in Table 2.

Except for YOLO, all of the models in Table 2 exhibit outstanding accuracy. InceptionV3 and MobileNetV2, out of all the pretrained models, have consistently produced smooth results from the start and had nearly the highest accuracy of all the other research. As seen in this study, when compared to other articles, InceptionV3 and MobileNetV2 have offered smooth accuracy per epoch, as seen in this study. VGG19 provided 92.82% accuracy as well, while the referenced article [62] used VGG-16 and obtained 95.9% accuracy. The accuracy of the referenced InceptionV3 and MobileNetV2 articles was 95% and 97.4%, respectively. InceptionV3 and MobileNetV2, on the other hand, were determined to be accurate to the tune of 96.92% and 98%, respectively, in this investigation. MobileNetV2 obviously outperforms these pretrained and custom models in terms of precision, recall, and F1 scores.

## 4. Conclusion

In this study, deep transfer learning models were given, one of which was fully customized. The remaining three models, MobileNetV2, VGG19, and Inceptionv3, are pretrained and adjusted. Models in this category and the correctness of the paper were nearly identical. There are 1,142 COVID-19 and 4,237 pneumonia chest X-ray pictures in the collection. The pretrained model has a 98% accuracy rate, while the customized deep transfer learning model has a 97% accuracy rate. Research on a larger data set and with additional pretrained models will be conducted in the future. In regards to our data set, these models have shown excellent outcomes. With these data sets, MobileNetV2 and VGG19 have done exceptionally well. To improve the picture quality, we first used the dynamic histogram equalization (DHE) method. This method has the potential to improve contrast enhancement without causing issues such as checkerboard effects or visual washout. Next, we built a simple VGG-based CNN model with only six layers, including ReLU activation, drop operation, and max-pooling layers, to recognize edges from original photos or previous feature maps. The findings demonstrate that our suggested model outperforms state-of-the-art CNN model designs, with an accuracy rate of 98%. Numerous assessments of various parameter shapes and loss functions were presented to demonstrate the efficacy of our proposed approach. Feature extraction and categorization worked effectively, and model verification confirmed that the findings were valid. In the quickest way possible, these models can detect COVID-19 and pneumonia using a simple chest X-ray image. X-ray technology is now available and is also cost-effective. As a result, it may be a very effective method of detecting COVID-19 and pneumonia. This method of testing and tracing the virus will be quick, with no threat of being stuck in a line and spreading the virus. This breakthrough will have a significant impact on the medical field. Using this method, COVID-19 and pneumonia patients can easily determine which factors can be attributed to the current global pandemic situation. A chest X-ray is comparable to collecting samples from the patient's nose in terms of safety. This type of technology will be beneficial to humanity in the years ahead. COVID-19 detection methods based on deep learning can be very useful in the present situation, considering the high number of patients.

## Figures and Tables

**Figure 1:** X-ray of COVID-19-affected chest.

**Figure 2:** Pneumonia-affected chest X-ray.

**Figure 3:** The proposed system.

**Figure 4:** System architecture (this figure is reproduced from Ziyang Zhao et al. [56], escalate).

**Figure 5:** The pretrained model's system architecture.

**Figure 6:** Training accuracy versus validation accuracy.

**Figure 7:** Training loss versus validation loss.

**Figure 8:** Training and validation AUC.

**Figure 9:** Confusion matrix.

**Figure 10:** COVID-19 prediction.

**Figure 11:** Pneumonia prediction.

**Table 1:** Comparison of experimental models.

No.	Configuration	Weighted F1 score (%)	Accuracy (%)
1	VGG-19	92.74	92.82
2	InceptionV3	96.0	96.92
3	EffNet threshold	94.68	94.95
4	MobileNetV2	98.0%	98.0%

**Table 2:** Model comparison.

This paper (model name)	Accuracy (%)	Reference paper (model name)	Accuracy (%)
VGG-19	92.82	Ref [12] (YOLO)	91.0
Inception V3	96.92	Ref [65] (Inception V3)	95.0
EffNet threshold	94.95	Ref [66] (VGG-16)	95.9
MobileNet V2	98.0	Ref [61] (MobileNetV2)	97.4

## Data Availability

The data utilized to support this research finding are accessible online at https://www.kaggle.com/tahiatazin1510997643/covid19-and-pneumonia-classification-dataset
